# Machine Learning for Smart Environments in B5G Networks: Connectivity and QoS

**DOI:** 10.1155/2021/6805151

**Published:** 2021-09-18

**Authors:** Saeed H. Alsamhi, Faris A. Almalki, Hatem Al-Dois, Soufiene Ben Othman, Jahan Hassan, Ammar Hawbani, Radyah Sahal, Brian Lee, Hager Saleh

**Affiliations:** ^1^Athlone Institute of Technology, Athlone, Ireland; ^2^Ibb University, Ibb, Yemen; ^3^Department of Computer Engineering, College of Computers and Information Technology, Taif University, P.O. Box 11099, Taif 21944, Saudi Arabia; ^4^Department of Electrical Engineering, Ibb University, Ibb, Yemen; ^5^PRINCE Laboratory Research, ISITCom, Hammam Sousse, University of Sousse, Sousse, Tunisia; ^6^Tunisia and School of Engineering and Technology, Sharda University, Greater Noida, India; ^7^Central Queensland University, Sydney, NSW 2000, Australia; ^8^School of Computer Science and Technology, University of Science and Technology of China, Hefei, China; ^9^School of Computer Science and Information Technology, University College Cork, Cork, Ireland; ^10^Faculty of Computers and Artificial Intelligence, South Valley University, Hurghada, Egypt

## Abstract

The number of Internet of Things (IoT) devices to be connected via the Internet is overgrowing. The heterogeneity and complexity of the IoT in terms of dynamism and uncertainty complicate this landscape dramatically and introduce vulnerabilities. Intelligent management of IoT is required to maintain connectivity, improve Quality of Service (QoS), and reduce energy consumption in real time within dynamic environments. Machine Learning (ML) plays a pivotal role in QoS enhancement, connectivity, and provisioning of smart applications. Therefore, this survey focuses on the use of ML for enhancing IoT applications. We also provide an in-depth overview of the variety of IoT applications that can be enhanced using ML, such as smart cities, smart homes, and smart healthcare. For each application, we introduce the advantages of using ML. Finally, we shed light on ML challenges for future IoT research, and we review the current literature based on existing works.

## 1. Introduction

The Internet of Things (IoT) ecosystem combines heterogeneous devices ranging from smartphones to connected cars, Unmanned Aerial Vehicles (UAVs, a.k.a. drones), sensors, robots, smart wearable devices, etc. Such massive and diverse IoT devices can lead to a high communication traffic load. Therefore, IoT demands high data rates, ultrareliable high Quality of Service (QoS), and low latency in real-time and high dynamic environments [1]. For instance, UAVs play a vital role in delivering services and keeping connectivity over smart city applications [2–4], such as monitoring traffic [5], public safety, disaster management, gathering data from IoT, and delivering wireless power to IoT devices. While IoT devices are distributed in robots for guiding robots to perform their task efficiently while collecting data of the surroundings, the Internet of Robotics Things (IoRT) represents a new version of IoT [6–8]. Furthermore, smart wearable IoT devices are distributed in the human body for healthcare monitoring in smart homes and smart healthcare applications. In the future of the IoT revolution, big data must be collected, sent to a massive number of IoT devices in real time with high dynamic environments, and intelligently analyzed for appropriate decision-making and producing accurate results. The appropriate decision-making criterion plays an essential role in conceiving and guiding IoT devices in several applications and services in real time. Gathered data in real time requires an efficient analytics technique to be predictive, descriptive, and adaptive. Classification of information and making an appreciated decision are creating the desired action in dynamic environments. For enhancing life quality in smart cities, intelligent techniques make IoT a worthy paradigm.

The recent communication technology (i.e., the fifth generation (5G), the sixth generation (6G)) plays a critical role in enhancing the massive Device to Device (D2D) communication. D2D communication requires intelligent functions to enable the IoT end devices' network improve the QoS and reliability efficiently [4, 9–13]. The intelligent functions for IoT services have to exploit the dynamic communication technology resources, gathering data to enhance the connection between devices efficiently and adaptively with high QoS and in real time. Artificial Intelligence (AI) has created opportunities to make machines or devices behave like humans to dynamically adapt IoT functions to keep the performance levels with changing context. AI can realize a reliable solution for devices to perform complex tasks effectively and efficiently, such as Artificial Neural Network (ANN). Recently, Machine Learning (ML) has been shown to provide self-learning [14, 15], self-organizing [16], self-optimization, self-reproducing [17, 18], and self-healing solutions for a broad range of IoT challenges. Moreover, ML and IoT are two cornerstone technologies enabling green public services at a lower cost and interacting with each other into an essential ecosystem.

This ecosystem realizes the promise of IoT requiring combination with an equally powerful and descriptive set of technology categories, such as ML. ML plays a pivotal role in QoS enhancement and connectivity between IoT end-to-end (E2E) devices for the provisioning of smart applications. ML assisting IoT enables green, public services at a lower cost in smart cities. ML is a promising technology to extract accurate and valuable information from IoT devices. Since the IoT devices have limited capability of processing, ML techniques will help optimize IoT network performance. Indeed, ML is undoubtedly the primary vessel carrying AI to investigate its use across many applications [19], including robotics, smart devices, smart industries, computer vision [20], smart processing, IoT devices connection, and autonomous systems. ML also plays several roles in big data analytics from multiple IoT devices in the IoT network, for example, in the deployment of the UAV for collecting data, mapping images of different IoT sensors in the UAV coverage area.

ML can play a vital role in redefining the physical layer functions such as modulation [21], coding and decoding [22], transmission, and reception for keeping the connectivity between IoT devices and UAV [21, 23]. First of all, researchers have often introduced ML techniques such as Deep Learning (DL) for communication [21, 24], resource availability and allocation [25], and control traffic [26]. However, the studies of [27, 28] mainly restrict their scope to Wireless Sensor Networks (WSNs) and Machine-to-Machine (M2M) connection [11, 29–31]. Hence, they do not mention the applications in which ML can be used for enhancing future networks. Moreover, the work reported in [29, 32] introduced the idea that connection and data collection of IoT devices are highly qualitative, but they did not provide a quantitative description of the ML for IoT connections. The authors in [33] focused on DL for the Internet of Multimedia Things (IoMT), including traffic management, parking, and security, to enhance smart city environments.  Figure 1 shows the potential applications of ML for achieving smartness in various aspects of IoT: energy, routing, living, industry, and everywhere.

The authors of [34] provided an overview of intelligent IoT and described the integration of ML and IoT. In addition, they discussed the idea of cognitive computing in several aspects, such as cognitive devices, cognitive networks, and cognitive analytics. Moreover, the study in [35] introduced computational intelligence in IoT for maximizing energy efficiency. It also explored IoT and cloud computing based on the environment.

The smart city is a complex ecosystem in which many advanced communication technologies, such as IoT and ML, are used to enable the smart city to be smart: clean, sustainable, and improving the life quality for residents [1]. The concept of smart cities refers to the smart application that helps fulfill city resource management purposes, improve QoS, and gather valuable information. These purposes are critical technology for reducing the cost and achieving managerial decision-making. The smart city consists of several applications such as smart healthcare, smart traffic, smart home, smart industries, smart building, smart parking, smart infrastructure, and smart monitoring.

Finally, the preliminary literature on ML for IoT such as [21, 29, 32, 36, 37] is dispersed, making it complicated to realize the ML for IoT due to a lack of common understanding. There is a gap in the thorough knowledge that can explain how to develop ML solutions to enhance IoT potential connectivity, reliability, QoS, and beyond. Thus, the main contribution of this paper is to present a systematic review of current literature and emerging work for IoT, which addresses the challenges and opportunities in developing ML for enhancing the capability of IoT devices to be smart in connection, security, reliability, and reliability of QoS and latency. We emphasize the use of using ML techniques to improve the IoT in real time and make the world smarter and greener.

### 1.1. Related Surveys

To the best of our knowledge, there does not exist a survey dedicated to reviewing the convergence of ML and IoT for enhancing the connectivity and QoS in IoT environments. However, particular studies exist on the use of ML techniques for IoT applications in dynamic environments. The authors of [27, 38–40] provided a survey of ML techniques for WSNs. They focused on ML techniques in WSNs for location, routing, clustering, security, and QoS. Furthermore, the authors reviewed several ML techniques for the infrastructure of WSNs, while our survey is not dependent on IoT infrastructure. The work presented in [41] reviewed different techniques of DL for IoT big data. It addressed different DL techniques to facilitate the learning and desired analytics in IoT applications. Several existing works are done based on ML for IoT in several applications [36, 37, 42–44]. Nonetheless, the authors did not cover all ML techniques for IoT; they only focused on DL for IoT big data. Furthermore, Perera et al. [45] reviewed and discussed the potential of using different ML techniques for context-aware computing in IoT. Fadlullah et al. [46] introduced DL techniques for traffic network control. They focused on network infrastructure; the work is different from our work that focuses on the convergence of ML for IoT applications based on connectivity and QoS.

### 1.2. Contributions

This survey is intended for IoT developers and researchers interested in making IoT applications smarter by using ML. The contributions of this survey are summarized below:

1. We survey ML techniques for convergence of IoT connectivity and reliability. This is, in contrast, compared to some surveys that introduced ML for IoT big data and data analytics, i.e., for specific IoT application domains. We also provide a comparison between different ML techniques for smarter IoT applications.
2. To adopt ML techniques in the IoT ecosystem, we select key features, challenges, and open issues of smart IoT applications. We reviewed all of the techniques and approaches for deploying ML for smarter IoT applications. Then, the future research directions and challenges for fruitful convergence of ML and IoT applications are highlighted.

### 1.3. Scope of the Study

ML techniques play a critical role in improving training and prediction to enhance accuracy. In this survey, we review the convergence of ML for enhancing connectivity and QoS in IoT environments within B5G networks. This survey focuses on the confluence of ML and IoT emerging technologies. However, this survey does not cover the details of the IoT network QoS and connectivity perspective.

### 1.4. Paper Structure

The rest of the paper is organized as follows, as also shown in Figure 2. In Section 2, we highlight IoT connectivity and reliability.  Section 3 presents the overview of ML. It includes a brief description of ML techniques such as Supervised Learning (SL), Unsupervised Learning (UL), and Reinforcement Learning (RL). ML for IoT applications in different domains is discussed in Section 4.  Section 5 explains the works that investigated ML for enhancing connectivity in IoT environments.  Section 6 reviews the works that incorporate ML to enhance QoS in IoT environments.  Section 7 discusses the ML for IoT applications. Future research directions and open issues are presented in Section 8. The paper is concluded in Section 9.

## 2. Internet of Things

IoT has reduced an enormous amount of human effort in almost all sectors. Trillions of machine-type devices such as connected vehicles, wearable sensors, or mundane objects will be connected to the Internet, forming a massive IoT ecosystem [47]. IoT is enabling devices to connect over wireless networks and collect data and process it in real time. IoT applications in smart cities include smart homes, smart grids, smart agriculture, smart healthcare, and smart streets and parking. However, to fulfill smart city applications, IoT is still facing many challenges such as computation, transmission capability, local data analysis in real time, end-to-end (E2E) latency, massive device connectivity, and privacy. Moreover, the available resources and energy of IoT devices are limited.

IoT applications are exponentially growing, e.g., smart homes [48], smart cities [49, 50], smart healthcare [51, 52], smart transportation [53, 54], smart agriculture [55], and smart street. The main essence of these applications is to make the machines smarter for prediction and data analytics, leading to smarter decision-making in smart environments. ML plays a vital role in enhancing IoT applications and represents the revolution of smart IoT technology to realize such smart environments.

## 3. ML Overview

ML was born and developed to allow machines to act intelligently, learning from their environments. Specifically, ML allows machines to learn from previous experiences autonomously using existing datasets, build suitable models to predict future behaviors and actions, and make intelligent decisions, as discussed in [19, 27, 56, 57]. ML is typically classified into Supervised Learning (SL), Unsupervised Learning (UL), and Reinforcement Learning (RL), as shown in Figure 3. SL is applicable for labeled input and output data. In contrast, RL is trained in the environment with data available in it. It aims to learn an environment and determine the suitable techniques in different environments. It is mainly used for robotics, navigation, and gaming [58]. Moreover, ML techniques have specific requirements for training data [59, 60]. ML can build regression to find the relationship between variables, classify unlabeled datasets, and cluster the data into different groups [61, 62].

ML techniques have become ubiquitous due to data collection, data analytics, IoT connections, smart devices, and the smart world [63]. Therefore, they provide great utility in different sectors and applications such as government, marketing, price stock, financial services, healthcare, smart things, robots, developing technologies, and dynamic environments. Furthermore, ML techniques are used to build a model which predicts dynamic environments and human behavior. Therefore, intelligent devices, machines, or robots can take intelligent actions and appreciate appropriate decisions according to the dynamic environments without human intervention. For instance, ML techniques help in real-time analysis of the data collected by IoT devices. ML training plays a crucial role in enabling ML to achieve the goal and discover the relationships between input and output data [24]. SL, UL, and RL pave the path for a bright future of machines that may eventually aid humans in doing routine activities.

### 3.1. Supervised Learning

It is a subset of the family of ML algorithms that are mainly used in predictive modeling. The majority of practical ML uses SL. It is named SL because, as illustrated in Figure 4, an algorithm learning from a training dataset may act as a teacher overseeing the learning process. As a result, a predictive model is one that is built using an ML approach and features or characteristics from training data to predict a value based on the other values in the input data. Furthermore, SL tries to create a model with relationships between the output and the input features. Therefore, this model can predict the future output values for new data based on what was learned from the previous datasets. A model is trained by requiring it to make predictions and correcting them when those predictions are incorrect. The training process is repeated until the model reaches the appropriate degree of accuracy on the test data.

Nowadays, SL makes up most of ML being used by systems across the world. The main categories of SL include regression and classification. In regression, the model tries to predict a continuous output based on the input variables. However, in the case of classification, the model instead tries to predict results in a discrete output. In other words, it tries to map input into discrete categories. For example, if *X* represents the input variables and *Y* represents the output variables, the learning map model represents the function of input and output variables such as

(1) $$\begin{array}{c} Y=f\left(X\right), \end{array}$$

where the main importance of the model is to predict the output *Y* when we have new input data *X*.

The tasks of the predictive model involve the prediction of future values based on using other values in the dataset. At the same time, the learning techniques attempt to create and model the relationship between input and output datasets, as shown in Figure 5. The predictive model implies forecasting and predicting future events and past events in real time in dynamic environments. SL predictive models are used to properly construct how they intend to learn and what they need to learn. Therefore, they consist of output variables that are to be predicted from a given set of independent variables. Using this set of variables, the model could map inputs to desired outputs. The training process will continue until the model achieves the desired accuracy. SL includes algorithms such as regression, K-nearest neighbors (KNN), random forest, decision tree, and logistic regression.

Classification is used to categorize all the available data which can form the output. For example, a Support Vector Machine (SVM) is used for demographic data such as marital status, age, or gender. Here, SVM is used to define the linear decision boundaries. ML uses SL approaches on historical data to make cognitive decisions.

### 3.2. Unsupervised Learning

The systems do not care about the datasets in the UL process, and the process becomes a little trickier. In simple terminology, ML is blind when it goes into the operation. Therefore, ML works to recognize the classification problem by finding similarities between objects and cluster them together. Moreover, ML can recognize the mistakes, then learn from them, and finally make an appreciative estimation and accurate decision. In SL techniques, predictions play a significant role, whereas, in UL techniques, homogeneity within clusters and heterogeneity across clusters play a significant role, as shown in Figure 6.

### 3.3. Reinforcement Learning

RL is one of the ML techniques experiencing an increasing use and contributing significantly to the growth of ML usage. Because it provides software agents and devices with a large sphere of control over the optimal behavior within a context, RL is a spin-off of the UL notion. Given the present condition of the environment, it chooses the optimal course of action. However, RL allows an agent to learn like a person by attempting new things and gathering experience from the attempts [64].

RL techniques can help the devices to learn from their surrounding environments and make an appropriate decision, for example, for mobile robots or drones [63]. RL plays a vital role in adjusting drone flying path and location and predicting the number of users that can be served within a particular coverage area in dynamic environments, as shown in Figure 7.

One of the IoT features is the expected scale in terms of the number of devices. Therefore, the optimizing task of IoT sensors cannot be performed manually for thousands of IoT devices. For example, reducing the duty services and using solar energy for sensor devices represent the optimal techniques for saving energy. However, the duty services will not perform optimally when the solar energy is not available, e.g., at night and in the dark winter, since the lack of enough power could cause the sensors to shut down. Therefore, throughout the sensor's operation, smart sensors may have to make decisions and plan their actions regularly based on the environmental changes. ML techniques are used for estimation, clustering regression classification, etc., as shown in Figure 8.

## 4. Machine Learning for IoT

ML plays a vital role in creating self-managed IoT devices, including heterogeneous and distributed components of different environments [65, 66]. Moreover, automated ML is used to solve real-world applications' massive IoT data problems [67]. The proposed automated ML provided the ability to recognize various patterns from IoT data and determine the best analytic process for different data to achieve the goal. Furthermore, ML can be used for prediction, big data analytics, and enabling IoT devices to learn from the dataset collected from the environments [68, 69]. For example, ML can analyze and predict drone mobility for delivering services to any specific area and for rescue and relief tasks during a disaster [2, 70]. During a disaster, smart sensors and cameras will collect data and capture the area of interest. Based on the collected data, the drone will take the appropriate path and desired action. Space robots play a vital role in improving many smart applications and manage disasters, such as high-altitude platforms [71–73], tethered balloons [74–79], and drones [2, 80–84]. They can efficiently deliver communication services to unreachable areas, remote areas, and rural areas.

Such examples of ML assisting IoT in achieving smart environments are numerous. IoT devices can learn and predict various types of information of devices' locations and behaviors and adapt their operation to such behaviors [85, 86]. Therefore, they can intelligently reduce the data traffic during their connections. For smart cities, IoT devices and ML for optimized predictions are imperative. For example, in smart streets, smart IoT devices will collect and process data using ML to predict the traffic load in a different street location. Another example is smart dustbins; deployed IoT smart sensors will be a catch to the dustbin container, and based on the collected data by sensors, bin collector vehicles will automatically come and take the dustbin from the whole container to keep streets greener and smarter.  Figure 9 shows the processes involved in all these examples.  Figure 10 shows ML classification for IoT based on SL, UL, and RL.

IoT devices help societies (i.e., businesses, medicine and healthcare, agriculture, building management, green environment management, smart cities, and smart things) collect a significant amount of data [87, 88]. ML for IoT assists with its surpassing feature in maintenance, monitoring, prediction, detection, and vehicle telemetry. ML enables IoT to optimize anomaly monitoring, detection, predictive data trends and maintenance, streaming and visualization of data, multivariate analysis, and data clustering [89]. Furthermore, ML helps take a decision via providing accurate input. Therefore, the combination of IoT and ML is growing in the market with such robust understanding and capability for performing complex works [90].  Figure 11 shows the power of ML for solving IoT issues in many applications.

ML in smart IoT devices has recently moved forward from managing traditional repetitive tasks to changing the tasks according to the changing environments continuously. Moreover, ML keeps evolving to make IoT devices smarter. Therefore, ML is rapidly becoming indispensable to IoT challenge solutions. IoT core components include connectivity, robotics, sensor data, and drone, which will lead to a requirement to be intelligent. For example, IoT needs smart devices to perform complex smart tasks; then, ML must help machines or devices learn from their environments and perform tasks [91, 92]. As a result, the smart sensor manifests the combination of ML and IoT in many successful integration technologies.

The IoT cloud allows things to connect anytime, anyplace, using any service, to anyone and anything. As things are connecting in the IoT cloud, the connection capabilities of a massive number of autonomous IoT devices are expected to grow significantly. The growth may lead to congestion during the channel access phase if a massive number of IoT devices access the channel, which leads to significant delay [93]. Therefore, numerous proposals for controlling the load of the random-access channel have been proposed [94–97]. These studies are mainly based on channel access probability. However, Kim and Kim [98] proposed DL to achieve efficient load-balancing in IoT.

The use of DL was proposed for heterogeneous data processing, vehicle platoon control, path planning, predicting driver behavior, and security to reduce the cloud's communication traffic load and computational load [99, 100]. DNN is ANN with multiple hidden layers in which the hidden layer will train based on the previously hidden layers [24]. It is suitable for recognition and implements the complex model's features based on massive datasets collected from IoT devices in smart cities. Furthermore, it has been applied in many research fields for significant improvements, such as big data, IoT, and speech recognition [24]. Long short-term memory (LSTM) is one of the most comprehensive methods of DNN used for sequence classification [101].

Authors in [102] provided an overview of DL techniques and applications in IoT. DL techniques are divided into four categories: convolutional neural networks, autoencoder, restricted Boltzmann, and sparse coding. These techniques are applicable and suitable for IoT applications such as image caption, visual tracking, and object detection. The DL techniques can learn hidden layer features; this made DL architecture more critical than other AI techniques [103]. DL is a subfield of ML, a subset of AI, as shown in Figure 12.

Data is helpful if it is actionable. IoT is about data, collection, detection, transmission, and so on, which can sustain IoT exponential growth in data volumes. To make the data actionable, data needs to be supplemented with creativity, context, and intelligent connectivity. Therefore, ML plays a vital role in IoT solutions based on enabling real-time responses and postevent processing. ML will enhance IoT application by predictive analytics, perspective analytics, and adaptive analytics. Smart sensors are used to provide real-time data and feedback, which enables three types of analytics: (a) predictive, (b) perspective, and (c) adaptive analytics.

### 4.1. Predictive Analytics

Predictive analytics is used for the tasks that involve predicting one value based on a given dataset of other values. In this case, the learning technique attempts to discover the relationship between the output values being predicted and the other features. The prediction is to imply forecasting past or future events. Predictive models, for example, may be used to regulate traffic lights in real time during rush hour. Predictive analytics can help the drone learn what it needs to know and how it should learn it. As illustrated in Figure 13, SL is a technique for training predictive models. The predictive model is trained until it reaches a specified degree of accuracy on the training dataset. Then, SL tries to optimize the model to identify the best combination of feature values that produce the desired output. The output values give a means for the drone to determine how effectively it is learning to do the required task (similar to supervision). Regression, decision tree, random forest, KNN, logistic regression, and other techniques are included in SL.

### 4.2. Descriptive Analytics

Descriptive analytics is used for tasks that benefit from the insight gained from summarizing data in valuable ways. It is also called pattern discovery which is used to identify valuable associations within data. The features have the same importance. It is called descriptive because there is no output to predict, estimate, or learn, and therefore the UL represents the training process. UL is a technique for dividing people into various groups, and it is commonly used to segment consumers into separate groups for targeted interventions. An Apriori algorithm and K-means, for example, are included in UL. Clustering is a descriptive analytics activity that divides a dataset into homogenous groups. It is sometimes used for segmentation analysis, which finds groups of people with similar characteristics.

Intelligent sensors can suggest immediate action at the edges of the events, thus avoiding outages and even disasters. In predictive analytics, the output of ML and DL is to predict future events and initiate proactive decisions without human intervention, as shown in Figure 14. For example, the autonomous car can reach its destination and select the best route based on traffic congestion and route optimization data. Prescriptive analytics is the final boundary of computational intelligence that will incorporate many applications such as health and prescriptive medical diagnosis and treatment, design manufacturing, stock market transactions, and power generation.

### 4.3. Adaptive Analytics

Continuous sensor data inputs can help systems learn how to execute the best actions on their own. Many airports and cities, for example, have self-driving monorail systems. For instance, nonrandomized database analyses are increasingly being used by healthcare decision makers to analyze the effectiveness, safety, and value of medicinal items. Data scientists in the healthcare field employ data-adaptive methodologies to enhance confounding control automatically. The advantages of data-adaptive analytic techniques to confounding correction in healthcare databases include data source independence, data-optimized covariate selection, and principled causal analyses using propensity score methodologies.

## 5. ML for Enhancing Connectivity in IoT Environments

M2M connectivity refers to machine communication without human interventions [104, 105]. It has been predicted that more than 15 billion M2M connectivity would occur via the Internet by 2021 [106]. These machines or devices would be connected, collect data from surrounding environments, and share collected data with each other and humans in high security. For instance, health sensors are used to collect data, securely send it to the end devices, and then transfer it to the cloud for seamless access by the specialist doctors [107], using asynchronous communication between applications and the cloud environment. Furthermore, blockchain and ML can secure data capture by robots and drones during disease breakout, as discussed in [108–110].

RL was proposed for connecting devices such as UAVs and investigating a trade-off between minimizing latency and maximizing the energy efficiency of the connection [111–114]. There are many benefits from increased revenues due to a combination of IoT devices and ML, such as IoT devices manufacturers, IoT data and information providers, and companies offering application services based on smart devices, as shown in Figure 15.

Recently, drones have become one of the IoT smart devices that play a vital role in enhancing connectivity and delivering data in real time [115]. Furthermore, the developments of 5G were based on the integration of drones as aerial base stations. Drone technology offers many advantages over terrestrial communication, such as dynamic deployment, low deployment cost, better channel conditions because of the Line of Sight (LoS), and spectrum efficiency [80, 82–84, 116]. Drones can function as a base station, relay station, and data collector [81, 117–120]. Drone data collection can replace many IoT devices in many applications such as agriculture, military, mining operations, and industrial inspection services, providing a greater flexibility of deployment with their flying capability. Here, intelligent self-organization techniques are required to optimize the flying path of drones. The authors of [70] applied ANN for optimizing drone position and trajectory based on signal strength. The drone can track users or any device's behavior in its coverage area and then collect data at any time in any place with any distance. The collected data will be analyzed using ML techniques. Due to the challenges of drone flight, such as limited battery capacity, drones are used for collecting data within a short period [121]. The authors in [122] proposed the DNN for image classification from gathered image data by drones. This work does not investigate the use of ML in the context of drones' wireless connection with each other or with IoT devices on the ground. This, however, is considered by authors in [123]. In this work, RL techniques can find the relationship between the data rate of each user and the location of the drone. The user mobility and content request distribution are used to predict the optimal drone locations.

Since the IoT devices are significantly increasing in number and are predicted to reach 100 billion devices in 2025 [124], the connectivity between devices via wireless networks and the Internet becomes a crucial success factor. Caching at the edge enables wireless network devices to reduce data traffic, store the most popular data in the close vicinity, and improve energy efficiency. Coded caching enables the network device to enhance bandwidth efficiency via coded multicasting transmission [125, 126]. However, network devices face many challenges, such as cache updating, cache placement optimization, and content popularity analytics. The authors in [127] combined computing and caching, which is used to store the most popular tasks.

Nonetheless, end-to-end latency minimization and energy consumption minimization are the challenges of optimizing mobile edge computing. Therefore, intelligent techniques are required for the prediction of mobile edge caching and computing. To this end, ML can be used to predict mobility patterns and users' content request distributions. For example, ML can be used to predict computational task requirements and users' interests by clustering the users with the same interests and storing the favorite contents. Therefore, predicting the tasks' computational requirements and user interests enables network devices to enhance connectivity and minimize global latency. Furthermore, the ML-based clustering algorithms can be used effectively to classify the users based on their interests and content request. The authors in [128, 129] proposed ANN to determine the cache replacement. However, the prediction of the content popularity is developed using the Hadoop platform [130].

Works in [131–134] discuss IoT device's connectivity and wireless communication using ANN. Here, ANN plays a vital role in enhancing the driver behavior modeling [131], classifying the objectives [133, 134], and predicting the speed of mobility [132]. Furthermore, IoT includes the increasing popularity of entities and objects that automatically transfer data over a network with unique identifiers. Growing the IoT communication comes from embedded sensors, computing devices, M2M communication, Vehicle-to-Vehicle (V2V) communication, smart grids, building and home automation, and smart wearable devices [135].

ML provides essential tools for IoT security. Many types of research have been conducted to identify IoT devices based on the signal properties, communication characteristics, and logical characteristics of network traffic [136]. For example, authors in [67] described a method for identifying rogue wireless devices and connecting the victim device to the network after being misled [137]. The authors of [138, 139] described techniques to cluster the network's traffic patterns associated with botnets in which exchanged data and device connection patterns are observed. Furthermore, ML is used to detect malware based on network traffic features [140, 141]. Authors in [142] introduce ML for IoT device identification based on network traffic, in which ML can help identify different kinds of nodes connected to the network. IoT device identification was based on data gathered from heterogeneous devices set and network traffic communication. In addition to work in [142], authors in [143] applied ML for IoT device identification based on IoT devices' classification into two categories based on energy consumption: high and low energy consuming devices.

Furthermore, [144] proposed a combination of k-means and SVM to identify the fingerprinting of smartphones by application behavior. They focused on smartphone feature classification and identified the time required for distinguishing smartphones. The authors of [145] applied ML techniques to identify application and traffic classification.  Table 1 summarizes the ML techniques for the identification and connectivity of IoT devices.

## 6. ML for Enhanced QoS in IoT Environments

Currently, in complex network and application environments of humans or things and robots communicating to each other and to the data center, different communication technologies need to cooperate for end-to-end QoS provisioning. The interaction between IoT devices is becoming a challenging issue, and improving the QoS in IoT networks is essential to the success of IoT applications [153]. Improving QoS plays a vital role in satisfying the users/things of services, for which the QoS techniques and parameters are discussed in [114, 154–160]. Due to the exponential growth of IoT devices, data collection, communication, and storage should be considered. Therefore, the study in [161] proposes IoT fog cloud, which plays a vital role in supporting the IoT services delay and QoS requirements. Then, the applications of ML techniques for IP traffic classification of IP networking to enhance the QoS were reviewed in [162]. The study focuses only on the IP traffic network and does not mention specifically the application of ML to the enhancement of the QoS of IoT devices. Furthermore, many studies have discussed the use of ML techniques to enhance the QoS, such as [163–168].

The study in [163] discusses the importance of using ML techniques in sensor intelligence routing and energy-aware routing for enhancing QoS. Authors in [166] focused on large-scale web QoS prediction based on Kernel ML (KML) for Industrial IoT. Integration of ML and IoT device connection will enhance the QoS and make smart, intelligent, and efficient things. ML can manage and operate the sensors optimally, as was shown in [169], where the optimizing ML techniques provided a role for balancing the required data rate and energy consumption of sensors.

Kumar et al. [170] developed a Bonsai algorithm for an efficient prediction on IoT devices locally without connecting to the cloud. In this scenario, ML plays an essential role in making efficient predictions locally, allowing the IoT device to work at any time everywhere, irrespective of the connection to the cloud. Therefore, it helps to reduce latency due to connection to the cloud, enhances bandwidth, reduces energy consumption due to data transmission to the cloud, extends battery life significantly, and enhances privacy. The authors in [171] applied ML-based data mining in smart cities where IoT constitutes information resources.

Along with the fast development of IoT technologies, the demand for high QoS, connectivity, and reliability is increasing exponentially. Combining ML and IoT will improve the QoS and make smarter, intelligent, and efficient devices or machines. Data can be collected as time-series data from IoT devices such as sensors. ML-based reinforcement and predictive techniques are more suitable for IoT datasets. ML and optimization schemes have not been sufficiently investigated from the perspective of IoT data and QoS.  Table 2 summarizes the ML techniques for improving IoT QoS.

The ML and IoT interdependence is poised to create a greener and smarter world. ML completes the vision of IoT being self-sufficient. IoT is used to collect data in real time, while ML can cause IoT devices to achieve fast processing and make decisions for any necessary action. Recently, the evolution is seeing ML application progress from assisted intelligence to augmented intelligence and ultimately autonomous intelligence, as shown in the Table 3. Furthermore, ML techniques for IoT in many applications are summarized in Table 4.

## 7. ML for IoT Applications

The combination of IoT and ML plays a vital role in real-time applications such as smart homes, smart cities, smart healthcare, smart grid, smart agriculture, smart industries, and smart things. The combination of IoT and ML will reshape our society and business lives dramatically. Recently, adapters of ML have had tremendous benefits in terms of prediction and detection. ML represents the core part of smart city applications which have gained attention in the research and industry sectors, especially in the big data fields. Many works have been done in this regard, such as [45, 187–190]. The authors of [187] provided a prediction technique to forecast power production using ANN. Similarly, the same techniques are used for traffic light control in smart cities [188] and context-aware computing in IoT [45]. In smart-grid networks, ML can detect malicious events before they occur [189]. Furthermore, ML techniques have outlined many issues, such as prediction of resource usage, data traffic monitoring, estimation of task response times, and optimal scheduling [190].

IoT devices create big data from the surrounding environment, and ML plays a vital role in analytics, such as big IoT applications in smart cities [61]. Therefore, IoT and ML's function is to get rid of the correlated information and reduce the size of big data gathered by IoT in smart cities [27]. As a result, data transmitted from the IoT devices to the central base station will be processed more efficiently and at less cost [27]. However, ML techniques can play a vital role in developing predictive methods to mitigate the lack of radio resources in IoT [191] as well. ML for IoT is efficient and effective in IoT security techniques such as IoT device authentication [192] and static malware analysis [193]. Below, we discuss some examples of IoT applications that could benefit from using ML techniques.  Table 5 presents a summary of the CNN, RNN, and DBN for several applications.

### 7.1. Smart Home

Smart IoT devices such as sensors must attach to the home to increase safety substantially and reduce risks simultaneously, including flooding and fire. Smart sensors will help to bring down the operating costs, e.g., alerting consumers to the optimum usage of dryers, reducing home insurance costs, and improving energy efficiency. Cost reduction and resident comfort can also be enhanced by adjusting the temperatures accordingly (i.e., switching heating and air conditioning on or off at the right times to exploit off-peak rates) and enhancing the house experience (i.e., optimizing climate control to suit different individuals). Smart homes allow the monitoring and controlling of devices for safe and convenient living. For instance, in the smart home, thermostats keep us warm, save money, monitor the environment, treat the source of pollution, and give personalized heath tips by fitness wearables. To enhance security, ML techniques play a critical role in smart home ecosystems [194].

### 7.2. Smart Healthcare

Sensors and other smart IoT devices can track a variety of body activities and data to improve safety and health. Smart sensors, for example, can be used to track manual laborers' load-carrying capacity and posture. Therefore, they are assisting in the prevention of injuries, the reduction of workers' compensation claims, and the improvement of labor productivity. Smart IoT devices can track human habits to enhance happiness, and smart sensors can help with general health by, for example, monitoring blood sugar levels and administering insulin as needed. Wearables are monitoring body functions, motion, and environment. The authors in [102] illustrated the capability of IoT to provide better healthcare.

### 7.3. Smart Cities

A smart city is an IoT application that enables cities to remain clean, sustainable, and efficient, improving the quality of life for citizens [195]. For example, DNN-based RL plays a vital role in controlling the streetlights to reduce energy consumption, adjust the signals dynamically, and prevent a collision. However, ANN has been used to solve several problems in smart cities with the help of IoT devices, such as urban traffic flow prediction [196] and parking availability prediction [197], as well as water demand prediction [198].

Integration of ML and IoT provides significant assistance in personal applications such as parking, medical assessment, energy saving, and future planning. For example, in parking, IoT assists in determining the suitable place for car parking spot based on traffic information, public parking sensor data, historical data, etc. Furthermore, ML in medical wearable devices can determine the status of the patient based on the symptom descriptions, measuring data from the body, medical records, and medical databases. In smart homes, based on the people's behavior inside the smart home, the smart devices (lamps, weather sensors, gate sensors, doors, etc.) will be turned on or off for energy saving. The ultimate aim of a smart city is to improve citizens' life quality, attain a sustainable environment, and reduce the cost of living. Therefore, the smart city requires the maturity of essential components, like security and privacy, service discovery, dynamic resource provisioning, edge computing, and IoT-enabled configuration [195]. Therefore, technologies such as AI and IoT have the potential to transform cities into sustainable smart cities.

## 8. Future Directions and Opportunities

### 8.1. Future Directions

ML has a huge potential in various applications beyond the obvious ones. DNN-based RL technique can be applied for optimizing content delivery. In order to optimize content delivery and cache replacement, each action taken for the DNN-based RL technique have to contain content delivery and one cache update technique. Therefore, DNN techniques are suitable for cache update techniques and storing large amounts of data. Furthermore, RNNs can be used to predict and estimate the demands of computational resources for each object.

ML techniques are an essential tool for addressing the challenges in drone connection. Different ML techniques can be suitable for various drone applications. For example, DNN-based RL can be used for interference control, power control, resource allocation, and user association. In particular, DNN can be used to improve the performance of network connections by optimizing resource allocation. Furthermore, RL technique can be used to predict the time duration for the drone to deliver service to the user or IoT devices on the ground. DNN-based RL can also store big data. Therefore, it can be used to store historical data of users and predict their locations. Moreover, DNN can be used for predicting path planning and data classification.

Higher accuracy requires higher energy and computation. The trade-off between the computation and energy requires training ANNs, and the learning technique provides the system's accuracy. However, data collected by IoT contains errors and has a different structure. Thus, we should know how to deal with and classify the data accordingly when we plan to train ML models using ANNs.

ML techniques are undoubtedly playing an essential role in solving several issues of IoT, especially in the case of smart operation and big data analytics. For example, Fuzzy Neural Networks (FNNs) can optimize IoT connections and map other systems that support smart city applications. Moreover, ML can be used for data recovery and compression to reduce latency and size of transmitted data. ML can extract the essential features from compressed data. On the other hand, DL can be used for recovery and data compression of the spatial domain such as CNN due to being effective in extracting features and patterns from big data, while RNNs can do data recovery and compression in time domains due to being suitable for relationship extraction in the time domain. Furthermore, DNNs can be used for IoT ecosystem identification and computational resource of IoT devices because DNN has multiple hidden layers related to IoT devices.

### 8.2. Opportunities

ML requires an extensive dataset such as locations of the IoT devices and the corresponding devices for enhancing the performance in real time. This may be considered as one of the ML limitations in IoT [27]. The dataset should be processed quickly in real time to make the IoT devices learn the dynamic environment. IoT devices' storage capacity may not be enough to store and process vast data [218]. Furthermore, the IoT devices can label the data autonomously and correctly [61] and their learning can be already done a priori. ML has also been implemented in the IoT as a centralized framework [27, 176], due to the limitation of resources at the IoT devices. The centralized cloud process is used to implement an effective ML. Hence, cloud-based processing will allow the IoT to use ML algorithms for big data analytics [61], where local storage and processing are prohibitive. However, designing a scalable wireless architecture with a large number of collaborating wireless access points, developing improved antenna technologies to improve throughput and reliability, and maintaining data confidentiality and security are all difficulties [29, 177] in achieving this. The importance of using cloud-based processing is to reduce communication overheads during the social correlation of data traffic and to increase energy efficiency [177, 178].

The most crucial advantage of ML techniques is their ability to predict, extract, classify, and characterize the regular pattern of massive datasets [219–221]. ML techniques can capture the nonlinear and highly dynamic relationship between input and output; they achieve the proper classifications, predictions, regression, clustering, and pattern recognition. Moreover, fuzzy approaches are used for controlling and designing a nonlinear system [72, 222, 223]. Recently, ML has attracted significant attention in smart IoT devices and has significantly influenced how humans interact with the developments of IoT devices and smart things [29, 32, 34, 224–226]. For instance, IoT devices are distributed in cities to make them greener and smarter [227]. Therefore, ML can predict pollution, road traffic control, smart house, smart parking, and smart street to reduce the congestion and achieve an energy-efficient, green environment. Here, the smart sensors will generate a massive dataset captured from environments, and the dataset can be stored and sent to another device to optimize its resources usage, monitor the pollution for green environments, and deliver smart services such as using drones for intelligent transportation in case of, for example, emergency and healthcare. ML can be helpful in making decision from different data from multiple sensors, thus facilitating more complex applications of IoT. In this case, using ML for optimized predictions becomes imperative. In a self-organizing context, RL can be used by IoT devices to learn and make an intelligent decision according to the situation of the environment [228]. For instance, RL is utilized for adjusting the UAV location and optimize the total number of IoT devices and users that can be served in a particular coverage area by the UAV.

In everyday living, the government and many companies are using ML and IoT for managing traffic, healthcare, environments, etc. On the other hand, IoT application is suitable for smart homes. Many IoT devices are designed to make homes smarter and greener, such as a smart lamp and smart sensors for temperature, humidity, heat, and heart rate monitoring. In addition, IoT devices such as sensors on the street can gather real-time data traffic conditions in smart streets and parking lots. Here, ML plays a vital role in developing a model based on the collected data. The created model can be used to predict the future and past events based on the experience data. Furthermore, the combination of IoT and ML can play a critical role in improving the precision of Google maps, traffic routing, and traffic prediction systems.

## 9. Conclusion

The presence of IoT is increasingly becoming ubiquitous in our living environments, with its sophisticated capability of detection, actuation, communication, identification, sensing, and control. The combination of ML and IoT devices plays a vital role in saving time and improving life quality with optimized traffic and reductions of pollution and energy consumption. This paper has provided a comprehensive survey focusing on ML and its potential applications in enhancing the connectivity and QoS of IoT devices. First, we have provided a thorough overview of analytics techniques of ML to facilitate the learning process for the IoT devices. Next, we have discussed the potential of using ML techniques to achieve the analytics in IoT collected data and applications, and then ML's promises and challenges have been introduced. ML implementation techniques for supporting IoT applications are discussed. We have reviewed the recent literature to include a state of the art technology in each of these sections. Finally, we shed light on the challenges and applications of ML for future IoT research, along with opportunities.

## Figures and Tables

**Figure 1:** Use of ML in IoT.

**Figure 2:** Paper structure.

**Figure 3:** Machine Learning (ML) classification techniques.

**Figure 4:** Supervised learning (SL).

**Figure 5:** Prediction mechanism workflow using SL.

**Figure 6:** Unsupervised Learning (UL).

**Figure 7:** Reinforcement Learning (RL).

**Figure 8:** ML techniques exploited for solving IoT issues.

**Figure 9:** ML automation and complexity level.

**Figure 10:** ML classification for IoT.

**Figure 11:** IoT cases solved with ML.

**Figure 12:** AI, ML, and DL.

**Figure 13:** Predictive analytics.

**Figure 14:** Descriptive analytics.

**Figure 15:** Combination of IoT and ML.

**Table 1:** ML-based identification and connectivity of IoT devices.

Ref.	ML techniques	Features	Highlights
[142]	Classification	➢ Device identification based on network traffic	✓ Identifying different kinds of nodes connected to the network
		➢ Distinguishing between IoT and non-IoT devices connected to the network	
[122]	DNN		✓ Classifying the images collected by the drone
[146, 147]	BPNN	➢ Failure detection	✓ Detecting sensor failure in IoT network
[148]	DNN and FNN	➢ Human activity classification	✓
[149]	ANN	➢ Tracking accuracy	✓ Improving IoT network tracking efficiency
[150]	CNN	➢ The accuracy of detecting images	✓ Enhancing the image detection accuracy of the IoT network
[151]	Bayesian	➢ IoT device classifications	✓ Classifying visual size of everyday objects
[144]	KNN/SVM	➢ Network traffic	✓ Identifying smartphones
			✓ Traffic generated by applications' background activities
[152]	Random forestry	➢ Network traffic	✓ Identifying device types

**Table 2:** ML for enhancing IoT QoS.

Ref.	ML techniques	Optimized components	Features	IoT applications
[161, 172, 173]	R- learning	QoS metrics	To provide the ability to respond to IoT and be suitable for wireless communication operations with enhancing QoS	QoS optimizations
[174]	Bayesian	Battery charge and transmission power	To obtain energy-efficient IoT using adaptive ECG signal filtering	
[166]	KLMS	Missing web service QoS value prediction	To predict the missing QoS values for the Industrial IoT based KLMS technique	Web service QoS of Industrial Internet of Things
[163]	SOM and NN	Delay and energy consumption	To obtain an accurate way to route data through the network	Sensor intelligence routing, energy-aware routing, and IoT monitoring and activity recognition
[175]	ML	Traffic classification	To realize adaptive the traffic classification framework of different kinds of networks	QoS-aware traffic classification
[162]	ML review	Heavy operational load, packet lengths, delay	To classify the IP traffic in IP networks and also to classify unknown traffic using ML	IP traffic classification techniques
[171]	DL	Reducing process time	To apply ML techniques for management in smart cities where IoT constitutes information resources	QoS in smart cities

**Table 3:** ML application progress.

Machine intelligence continuum	Assisted intelligence	Autonomous intelligence	Augmented intelligence
Nature of tasks	No change	Change	Change
Automated	Tasks are automated	Decisions are automated	Machines' need for human guiding
Learning	Machines learn	Machines learn continuously	Machines learn and inform humans
*Examples*	Machinery, boilers, ovens	An autonomous vehicle, smart investment	A business strategy, analysis using Machine Learning, smart clinical decision support

**Table 4:** Summary of the ML techniques for IoT.

Category	Data type	Learning technique	Application in IoT
SL	• Predicting labeled data	Regression	Data compression and aggregation [176], big data analytics [27, 61, 177], and query processing [178]
	• I/P and O/P are known	K-nearest neighbor	
	• Regression	Support Vector Machines	
	• Classification	Bayesian learning	

UL	•Descriptive model, “unlabeled” data •Clustering and association	K-means	Heterogeneous networks [9]
		PCA	Smart grid [179]
		ICA	Spectrum learning [11]

RL	•Classification and control •Reacting to an environment	MDP/POMDP	Power control [180], energy harvesting [181], IoT radio recourses management [182, 183], energy efficiency scheduling [182], and use of a drones for enhancing communication [184]
		Q-learning	Small cells [185]
		Multiarmed bandit	D2D networks [186]

**Table 5:** CNN, DBN, and RNN used for supporting IoT application.

Technique	Features	Used	1	2	3	4	5	6	7	8
CNN	➢ Requiring a large train dataset	Traffic sign detection	[199]	[171]	[200]	[171, 201–203]		[204–206]	[207–211]	[212, 213]
	➢ Biggest part of computations									
	➢ Convolution layers									

DBN	➢ Discovering hierarchical features	Security threat identification	[98]	[98]			[214]	[215]		
	➢ layer by layer training network	Fault detection classification								

RNN	➢ Processing sequences data via internal memory	Behavior detection				[216]	[217]			
	➢ IoT with time-dependent data	Identifying movement pattern								

1: connection; 2: QoS; 3: smart home; 4: smart cities; 5: smart grid; 6: smart healthcare; 7: smart agriculture; 8: location.

## Data Availability

There are no relevant data to be made available.
